# Visual Analysis of Sports Actions Based on Machine Learning and Distributed Expectation Maximization Algorithm

**DOI:** 10.1155/2022/5640562

**Published:** 2022-06-25

**Authors:** Yan Luo

**Affiliations:** Jinhua Polytechnic, Jinhua 321000, China

## Abstract

In order to improve the scientificity of sports action analysis, this paper constructs a sports action analysis model based on machine learning based on the greedy algorithm and the bat algorithm. According to the structural characteristics of the model, the structure of the model is reflected in the form of face order, that is, the face neighborhood structure. Moreover, this paper judges the degree of similarity between model faces through the pros and cons of the order and applies it to the structural similarity matrix between models. In addition, this paper establishes corresponding mathematical models for the shape and structure of the model and constructs the shape similarity matrix, the surface neighborhood structure similarity matrix, and the structure similarity matrix between the source model and the target model. Finally, this paper designs and implements CAD model retrieval methods based on greedy algorithm and bat algorithm and designs experiments to compare the performance of the algorithm proposed in this paper with traditional algorithms. The result of the experiment shows that the algorithm proposed in this paper has obvious advantages in sports action analysis compared with the traditional algorithm.

## 1. Introduction

Scientific analysis of sports movements can effectively improve the effects of sports training, provide athletes with more scientific and effective training guidance, and reduce training injuries. Therefore, auxiliary sports training through intelligent sports movement recognition and analysis models is the direction of future sports training development. With the development of cost-effective sensors and the advancement of human body pose estimation algorithms, it has become easier to obtain three-dimensional and two-dimensional bone point data from human motion video data. The motion trajectory of the human skeleton points in the time sequence can represent the actions in the time sequence and is not affected by light, clothing, skin color, and so on. In recognition of the human body local limb movement with higher fine-grained requirements, the geometric characteristics between the bone points can be expressed naturally, and the movement has good interpretability. These characteristics make human action recognition based on skeletal point data an important direction in computer vision.

Action recognition based on bone points needs to design different classification algorithms according to different features of the extracted bone points. The relative motion of the human bones will produce the posture, so the relative position changes of the bone points can characterize the posture changes in the sequence. Moreover, the angle change of the connected bones indirectly reflects the change of the movement there. Therefore, the spatial structure used in this paper is the vector modulus ratio of the characteristic bone points and the vector angle of the bone points as the bone points.

Video retrieval is to search for useful or needed information from a large amount of video data. It is mainly based on the given example or the designed special diagnosis description to find out the video clips that meet the conditions in a large amount of video data. With the widespread use of video capture equipment, the amount of available video data is also increasing. If manual processing is used to process video data, it will cause a substantial increase in labor costs. However, if a computer is used instead of labor to analyze the human motion behavior in the video, it can avoid excessive labor costs. Moreover, it can be faster, more comprehensive, and accurate in the labeling and indexing of videos, thereby helping people find important information of interest more conveniently.

## 2. Related Work

Most feature extraction models describe a certain part of the model, and it is difficult to extract and describe all functional models. Some research proposed a 3D shape descriptor and weight combination optimization scheme and used it to retrieve CAD models [1]. This scheme judges the similarity between models based on the weighted sum of the *L*1 distance on the distance histogram corresponding to the descriptor and uses the weight combination optimization scheme to improve the retrieval accuracy of the 3D model database. Some research proposed three combined feature descriptors and one class-based feature descriptor and applied them to model retrieval [2, 3]. Some research introduced coupled machining feature clusters to represent the three-dimensional CAD model as a structured model with machining features as a carrier and uses multilevel feature descriptors to establish a machining feature similarity evaluation model. Some research used fuzzy clustering of some physical descriptors to generate a multiscale index of the 3D model database for fast matching.

Some research proposed an ontology-based 3D CAD model retrieval algorithm. The CAD model is divided into several related subcomponents, and semantic description and annotations are added to complete the similarity evaluation between the models. Some research used hierarchical feature ontology and ontology mapping to generate semantic descriptors based on semantic descriptors for ontology reasoning so that the retrieval system can obtain better performance [4]. Some research used the ontology to describe the functional semantics of the CAD model and semiautomatically annotated the functional semantics of the CAD model according to the attribute adjacency graph, thereby establishing a CAD model library that supports functional semantic model retrieval according to the existing model retrieval technology and feature extraction method [5, 6]. Some research used deep learning technology to train model features and built a deep neural network classifier for the three-dimensional computer-aided design model. Some research used another way to extract the feature vector of the three-dimensional model and to predict and match the model, effectively assessing the difference between the two models [7]. In addition, many researchers began to convert three-dimensional models into two-dimensional graphics to extract the edge and shape information of the model to describe the characteristics of the model. Some research divided the surface adjacency graph into convex, concave, and flat areas, used the area attribute code to represent the surface area, and compared the area attribute codes to measure the similarity between the models. Some research used B-Rep information and label attribute adjacency graphs to represent 3D CAD models and used a two-stage filtering strategy combined with graphic code indexing to construct filters and verification frameworks to speed up the retrieval of 3D models [8, 9].

Many researchers have also begun to use this framework to optimize and improve traditional machine learning algorithms. Some research has studied clustering algorithms under the Hadoop cloud platform [10]. Some research used the MapReduce distributed framework to parallelize the improvement of the traditional ant colony algorithm, which makes the traditional ant colony algorithm faster and more effective when processing large-scale data sets [11, 12].

Some research used Newton's method to solve the beta distribution parameter algorithm and proposed a suitable initial value selection algorithm to enable the EM (Expectation Maximization) algorithm to effectively solve the parameters of the implicit regression model. Some research proposed an EM algorithm based on density detection, which selected the initial value based on density and distance to reduce the influence of the traditional EM algorithm's initial value selection on the convergence effect [13–15]. Some research proposed a fast and robust finite Gaussian mixture model clustering algorithm and applied an entropy penalty operator to the mixing coefficients of the model components and the probability coefficients of the components to which the samples belong to make the algorithm converge to a certain value in a few iterations. Some research used the greedy algorithm method and set appropriate thresholds for the hidden parameters so that the traditional EM algorithm can obtain the number of model components of the Gaussian mixture model in a few iterations without presetting the number of model components.

## 3. EM Algorithm

The EM algorithm is an iterative method and is used to solve the maximum likelihood estimation or maximum a posteriori estimation of parameters in the probability model, which can greatly reduce the computational complexity of solving the maximum likelihood estimation. The specific algorithm flow is as follows.

If we assume that the sample set is *X*={*x*_1_, *x*_2_, *x*_3_,…, *x*_*m*_} and obeys the Gaussian mixture distribution, the probability density function *f*_*k*_(*x*) of the Gaussian mixture distribution is

(1) $$\begin{array}{c} f_{k}\left(x\right)=\sum_{j=1}^{k}w_{j}\Phi_{j}\left(x_{i};\theta_{j}\right). \end{array}$$

Among them, *x*_*i*_ is a P-dimensional vector, Φ_*j*_(*x*_*i*_; *θ*_*j*_) is the probability density of the *J*th Gaussian model component, and *θ*_*j*_ is its parameter. *w*_*j*_ is the mixing coefficient of the *j*th component, describing the proportion of the sample covered by the *j*th Gaussian model component to the total sample, and *k* is the number of model components of the Gaussian mixture model.

(2) $$\begin{array}{c} \theta_{j}=\left(\mu_{j},\sum_{j}\right). \end{array}$$

*μ*_*j*_ is the mean value of Gaussian model components, and ∑_*j*_ is the covariance matrix of Gaussian model components. Among them, the expression of Gaussian component probability density Φ_*j*_(*x*_*i*_; *θ*_*j*_) is

(3) $$\begin{array}{c} \Phi_{j}\left(x_{i};\mu_{j},\sum_{j}\right)=\frac{\exp\left\{-\left(1/2\right){\left(x_{i}-\mu_{j}\right)}^{T}\sum_{k}^{-1}\left(x_{i}-\mu_{j}\right)\right\}}{{\left(2\pi \right)}^{p/2}{\left|\sum_{k}\right|}^{\left(1/2\right)}}. \end{array}$$

The initial value *μ*_0_, ∑_0_, *w*_0_ is given, and steps *E* and *M* are repeated until the algorithm converges.

Step E: according to the initial value of the parameter *θ* or the parameter value obtained in the last iteration, the posterior probability of the recessive variable (i.e., the expectation of the recessive variable) is calculated as the current estimated value of the recessive variable:

(4) $$\begin{array}{c} Q_{i}\left(z^{\left(i\right)}\right)≔f\left(z^{\left(i\right)}|x^{\left(i\right)};\theta \right). \end{array}$$

Step M: by calculating the maximum value of the likelihood function, new parameter values are obtained:

(5) $$\begin{array}{c} \theta ≔\text{aeg}\underset{\theta }{\max}\sum_{i}\sum_{z^{\left(i\right)}}Q_{i}\left(z^{\left(i\right)}\right)\text{log}\frac{f\left(x^{\left(i\right)},z^{\left(i\right)};\theta \right)}{Q_{i}\left(z^{\left(i\right)}\right)}. \end{array}$$

Finally, the following results are obtained:

(6) $$\begin{array}{c} w_{k}^{t+1}=\frac{\sum_{i=1}^{n}f\left(k|x_{i},\theta^{t+1}\right)}{n},\\ \mu_{k}^{t+1}=\frac{\sum_{i=1}^{n}f\left(k|x_{i},\theta^{t+1}\right)x_{i}}{\sum_{i=1}^{n}f\left(k|x_{i},\theta^{t+1}\right)},\\ \sum_{k}^{t+1}=\frac{\sum_{i=1}^{n}f\left(k|x_{i},\theta^{t+1}\right)\left(x_{i}-\mu_{k}^{t+1}\right){\left(x_{i}-\mu_{k}^{t+1}\right)}^{T}}{\sum_{i=1}^{n}f\left(k|x_{i},\theta^{t+1}\right)}. \end{array}$$

Among them, *w*_*k*_^*t*+1^ is the *k*-th class weight, *μ*_*k*_^*t*+1^ is the *k*-th class mean, *θt*+1 is the *d*-dimensional vector, and ∑_*k*_^*t*+1^ is the *k*-th class covariance matrix.

Finally, through calculation, the parameter values of the Gaussian mixture model are obtained, and each sample is found in the subordinate class to obtain the final clustering result.

## 4. Greedy EM Algorithm

Based on the original probability density function *f*_*k*_(*x*) of the Gaussian mixture distribution of the EM algorithm, when a new component *δ*(*x*; *θ*) is brought into an existing k-component mixture density function *f*_*k*_(*x*), a new Gaussian mixture model density function is generated:

(7) $$\begin{array}{c} f_{k+1}\left(x\right)=\left(1-\alpha \right)f_{k}\left(x\right)+\alpha \delta \left(x;\theta \right). \end{array}$$

Among them, *α* is the mixing coefficient of the newly added model components, 0 < *α* < 1.

Then, the newly generated log-likelihood function is

(8) $$\begin{array}{c} L_{k+1}=\sum_{i=1}^{n}\log\left[\left(1-\alpha \right)f_{k}\left(x\right)+\alpha \delta \left(x;\theta \right)\right]. \end{array}$$

After the new Gaussian mixture model, including the mixture model components and the new components, is obtained, the mixture model *f*_*k*_(*x*) is set as unchanged. Therefore, the core of the greedy EM algorithm is to optimize the mixing coefficient *α* of the new model components and the parameters of the new components to calculate the highest value of the newly generated log-likelihood function *L*_*k*+1_. Therefore, we first find a set of initial parameters *μ*_0_, ∑_0_, and *α*_0_ of the new component through a global search. At *α*_0_, the second-order Taylor formula of *L*_*k*+1_ is expanded, and the quadratic function of *α* is maximized to obtain an approximation of the likelihood function:

(9) $$\begin{array}{c} {\hat{L}}_{k+1}=L_{k+1}\left(\alpha_{0}\right)-\frac{{\left[L_{k+1}^{\prime }\left(\alpha_{0}\right)\right]}^{2}}{2L_{k+1}^{\prime \prime }\left(\alpha_{0}\right)}. \end{array}$$

In the formula, *L*_*k*+1_′ and *L*_*k*+1_^″^ are the first and second differentials with respect to *α*. If we define

(10) $$\begin{array}{c} X\left(x;\theta \right)=\frac{f_{k}\left(x\right)-\delta \left(x;\theta \right)}{f_{k}\left(x\right)+\delta \left(x;\theta \right)}, \end{array}$$

then the log-likelihood local optimum of *L*_*k*+1_ near *α*_0_=0.5 can be written as

(11) $$\begin{array}{c} {\hat{L}}_{k+1}=\sum_{i=1}^{n}\log\frac{f_{k}\left(x_{i}\right)-\delta \left(x_{i};\theta \right)}{2}+\frac{1}{2}\frac{{\left[\sum_{i=1}^{n}\chi \left(x_{i};\theta \right)\right]}^{2}}{\sum_{i=1}^{n}\chi^{2}\left(x_{i};\theta \right)}. \end{array}$$

Thus, the formula for estimating $\hat{\alpha }$ of the newly added model components can be obtained:

(12) $$\begin{array}{c} \hat{\alpha }=\frac{1}{2}-\frac{1}{2}\frac{\sum_{i=1}^{n}\chi \left(x;\theta \right)}{\sum_{i=1}^{n}\chi^{2}\left(x;\theta \right)}. \end{array}$$

Thus, the estimated value of the new model component is obtained, and then the optimal solution {*α*_*k*+1_, *μ*_*k*+1_, ∑_*k*+1_} of the new model parameter is extracted through the formula iteratively to extract the log-likelihood function value *L*_*k*+1_ of the new Gaussian mixture model.

The actual processing process of MapReduce is

(13) $$\begin{array}{c} \text{Input}⟶\text{Map}⟶\text{ Sort}⟶\text{Combine}⟶\mathrm{Partition}⟶\mathrm{Reduce}⟶\mathrm{Output}. \end{array}$$

The specific workflow is shown in Figure 1.

For the Map phase, the algorithm begins to process data on the key-value pairs parsed in the Input phase. First, it initializes and then adds new model components to the single Gaussian mixture model initialized in each node. The new model component is a standard normal distribution with a mean value of 0 and a standard deviation of 1, and then the initialized mixing coefficient *α*_0_ of the new model component is obtained. Among them, the initial parameter value of the *l*th node model is

(14) $$\begin{array}{c} \mu_{0}^{l}=E\left(x\right),\\ \sum_{0}^{l}=\text{cov}\left(x\right),\\ w_{0}^{l}=1,\;1\leq l\leq h. \end{array}$$

Then, the new model component parameters *μ*_*k*_^*t*+1^ and ∑_*k*_^*t*+1^ of each node are calculated to obtain the new model component, then the new model component mixing coefficient *α*_*k*_^*t*+1^ is obtained, and the new Gaussian mixture model density function is obtained. The generated key value is used as the number of iterations, and the key-value pair with the Gaussian mixture model density as the value is output to the next stage.

Before output to the Reduce stage, there will be a series of intermediate processing. For the Sort stage, because the key value in the key-value pair is set to the number of iterations, this stage does not need to be considered too much. For the Partition stage, in this stage, the number of keys is the number of iterations, and the key-value pairs generated under the same iteration level have the same key value. Therefore, for each key-value pair generated in the Mapper phase, a Reduce job is assigned, the key and value values of the key-value pair are serialized into a byte array, and then the result is written into the buffer to wait for the call.

For the combine stage, the key-value pairs obtained by all nodes are integrated. Under the same number of iterations, the key values of the key-value pairs obtained from each node are the same, so the value values in these key-value pairs are integrated into a value set; namely,

(15) $$\begin{array}{c} \text{list}\langle \text{key,value}\rangle ⟶\langle \text{key,list}\langle \text{value}\rangle \rangle . \end{array}$$

Among them, key is the number of iterations, and value is the Gaussian mixture model density.

For the Reduce phase, the key-value pair generated in the combine phase is 〈key,list〈value〉〉. That is, the Gaussian mixture model density function set in the key-value pair is summed, then the logarithm is taken, and the integrated log-likelihood function is obtained as

(16) $$\begin{array}{c} F_{k+1}=\sum_{i=1}^{n}\text{log}\sum_{i=1}^{h}f_{k}^{t+1}\left(x\right). \end{array}$$

Then, it is judged whether *F*_*k*_ satisfies the convergence condition, and the judgment factor is set:

(17) $$\begin{array}{c} \lambda =\left|\frac{F_{k}^{t+1}}{F_{k}^{t}}-1\right|. \end{array}$$

When *λ* < 10^−6^, if the algorithm satisfies the convergence condition, the algorithm proceeds to the next step of judgment. However, if it does not converge, the algorithm restarts the maximum likelihood estimation operation.

For the Output stage, it is judged whether the convergence condition *F*_*k*_ satisfies *F*_*k*+1_ ≤ *F*_*k*_. If the convergence conditions are not met, new model components are added again. However, if the convergence condition is met, the output condition is met, and the result is output in the form of key-value pairs according to the format of the output file. If the value is *F*_*k*_ that satisfies the output condition, then the *k* value corresponding to *F*_*k*_ at this time is the number of output ideal model components. The final algorithm flowchart is shown in Figure 2.

## 5. Implementation of Distributed Greedy EM Algorithm

According to the programming model of MapReduce, corresponding functions are designed for program operation. In the realization of the distributed greedy EM algorithm, because the main process of the distributed greedy EM algorithm includes the reading of global data, the update calculation of Gaussian mixture model parameters, and the three aspects of iteration, the function design and implementation of these three main steps are carried out.

### 5.1. Reading of Global Data

In the algorithm of this paper, the data needs to be globally searched and initialized, and all the data in the distributed file system can be obtained through the setup function in the Mapper class. Since the distributed greedy EM algorithm needs to obtain global data variables after each iteration, it can be implemented through the setup function in the MapReduce programming model. For the distributed greedy EM clustering algorithm, the Map task is completed through each data node, and the parameter values of the Gaussian mixture model are obtained. The setup function can obtain data files stored in HDFS while ensuring that each data node shares the same variables. Because the global variables mentioned are sometimes required to be acquired and used, the Map function can be defined after the setup function is defined. First, the path of the model parameters of the distributed greedy EM algorithm is obtained and stored in the Configuration object. For the first iteration, the initial parameter values of the model are obtained from the path stored in the Configuration object. Then, when the subsequent iterations are performed, the output path is obtained from the Reduce function in the previous iteration.

Then in the Mapper class, the setup function is reassigned, and the corresponding data is obtained from the global file from the Configuration object. After the reading is completed, the parameter values are read into the cluster object through the Buffered Reader function, thus completing the reading of the global data.

### 5.2. Update of Gaussian Mixture Model Parameters

When the parameters are updated through the maximum likelihood estimation of the Gaussian mixture model, the parameters include the mixing coefficient, mean value, and covariance matrix of the new model components. Among them, the covariance matrix needs to obtain the mixing coefficient and mean value of the newly added model components. Therefore, two functions need to be designed to update them separately. The constant MapReduce function is defined to obtain the mixing coefficient and mean value of the new model components, and the matrix MapReduce function is defined to obtain the covariance matrix and output all parameter values.

For the constant MapReduce function, every time the mixing coefficient and mean value of the new model component are performed, all the parameter values obtained from the previous iteration (the mixing coefficient, mean value, and covariance matrix of the new model component) are required. Therefore, the data in the cluster global object is read in the step function. However, for the matrix MapReduce function, the mixing coefficient and mean value of the new model components obtained by the constant MapReduce function update this time are required. Moreover, the covariance matrix obtained this time will be used as the input of the constant MapReduce function of the next iteration, so it is necessary to use the step function to read the mixing coefficient, mean, and covariance matrix of the new model component obtained this time into the cluster_new object.

### 5.3. Iteration of Distributed Greedy EM Algorithm

When the distributed greedy EM algorithm is iterative, it needs to store the output result of the previous MapReduce in HDFS and use it as the input of the subsequent iterative MapReduce. Moreover, after an iteration is completed, the corresponding median data needs to be deleted. Therefore, the iterative process when designing the distributed greedy EM algorithm is shown in Figure 3.

Our work used the bat algorithm to find the optimal face matching sequence. In the process of bats searching for the structural similarity matrix FC of the source model and the target model, in order to make the bat move to the best position, a corresponding fitness value is set for each bat. The position solution sequence of the *i*th bat in the structural similarity matrix FC is (1, *j*(1)), (2, *j*(2)),…, (*i*, *j*(*i*)),…, (*m*, *j*(*m*)). Among them, *j*(*i*) represents the target face number *i*=1,2,…, *m* that matches the *i*th face of the source model. The calculation process of the fitness function of the *i*th bat is given, as shown in the following formula:

(18) $$\begin{array}{c} f\left(x_{i}\right)=\sum_{t=1}^{m}S\left[t,j\left(t\right)\right]. \end{array}$$

In the process of searching for the optimal solution, the points acquired by the bat are discrete. In a *d-dimensional* search space, the size of the population is *N*. *x*_*i*_ represents the position of the *i*th bat, that is, a two-dimensional sequence pair composed of the row and column indices of the structural similarity matrix, and *v*_*i*_ represents the flight speed of the *i*th bat. At time *t*, the speed of bat *i* is updated as follows:

(19) $$\begin{array}{c} v_{i}^{t}=v_{i}^{t-1}+\text{round}\left[\left(x_{i}^{t-1}-x^{*}\right)Q\left(i\right)\right]. \end{array}$$

Among them, round represents the rounding operation, and *Q*(*i*) is the frequency of the *i*th bat, as shown in the following formula:

(20) $$\begin{array}{c} Q\left(i\right)=Q_{\min}+\left(Q_{\min}-Q_{\max}\right)*\mathrm{rand}. \end{array}$$

rand is a uniformly distributed random number between [0,1], and *x*^*∗*^ is the current optimal position solution. Taking source model *A* and target model *B* as examples, using the above formula, a set of velocity solutions about the current *i*th bat can be obtained. From the sequence of these solutions, a set of sequence solutions is obtained to simulate the whole process of bats searching for the optimal position sequence.

A set of solution sequences are randomly obtained to represent the current optimal position solution *x*^*∗*^:

(21) $$\begin{array}{c} \left(1,2\right),\left(2,3\right),\left(3,4\right),\left(4,5\right),\left(5,1\right),\left(6,9\right),\left(7,8\right),\left(8,6\right),\left(9,7\right). \end{array}$$

The velocity solution sequence of the *i*th bat at *t* − 1 is

(22) $$\begin{array}{c} \left(1,6\right),\left(2,-2\right),\left(3,8\right),\left(4,0\right),\left(5,4\right),\left(6,-16\right),\left(7,-10\right),\left(8,6\right),\left(9,6\right). \end{array}$$

The velocity solution sequence of the current *i*th bat at time *t* can be obtained:

(23) $$\begin{array}{c} \left(1,8\right),\left(2,-3\right),\left(3,10\right),\left(4,0\right),\left(5,4\right),\left(6,-21\right),\left(7,-12\right),\left(8,8\right),\left(9,8\right). \end{array}$$

The speed of the *i*th bat at time *t* is *v*_*i*_^*t*^, and its position at time *t* − 1 is *x*_*i*_^*t*−1^. The calculation process of *x*_*i*_^*t*^ is as follows:

(24) $$\begin{array}{c} x_{i}^{t}=\mathrm{round}\left(x_{i}^{t-1}+x_{i}^{t}\right). \end{array}$$

Among them, round represents the rounding operation.

The position solution sequence of the *i*th bat at time (*t* − 1) is

(25) $$\begin{array}{c} \left(1,2\right),\left(2,3\right),\left(3,4\right),\left(4,5\right),\left(5,1\right),\left(6,9\right),\left(7,8\right),\left(8,6\right),\left(9,7\right). \end{array}$$

The position solution sequence of the *i*th bat at time *t* can be calculated:

(26) $$\begin{array}{c} \left(1,10\right),\left(2,0\right),\left(3,14\right),\left(4,5\right),\left(5,5\right),\left(6,-12\right),\left(7,-4\right),\left(8,14\right),\left(9,15\right). \end{array}$$

The obtained bat position solution sequence is processed, and the processing process is as follows:

*Step 1*. The remainder operation of the surface sequence (mod) is used to solve the situation that the second component of the bat position solution is out of bounds, and the position solution is obtained again.
The algorithm uses the following formula to take the remainder and reacquire the current bat position solution. Among them, mod is the remainder function.
  (27) $$\begin{array}{c} x_{i}^{t}=\text{mod}\left[x_{i}^{t},\left(m+1\right)\right]. \end{array}$$
The mod operation is used to update the position solution sequence of the *i*th bat at time *t*, and the result is
  (28) $$\begin{array}{c} \left(1,0\right),\left(2,0\right),\left(3,4\right),\left(4,5\right),\left(5,5\right),\left(6,8\right),\left(7,6\right),\left(8,4\right),\left(9,5\right). \end{array}$$
After the mod operation, the second component of the bat position solution may appear 0. If 0 appears, the algorithm executes Step 2; otherwise, the algorithm executes Step 3.
*Step 2*. The second component of the processed position solution is 0 (replace operation). The random sequence of the face number *m* of the source model is obtained, and the value of the second component that does not appear in the position solution after the remainder is found. After that, the found value is used to fill in the 0 in the second component of the position solution after the remainder.
The replace operation is shown in Figure 4. The black solid point on the left is the position solution sequence after taking the remainder:
  (29) $$\begin{array}{c} \left(1,0\right),\left(2,0\right),\left(3,4\right),\left(4,5\right),\left(5,5\right),\left(6,8\right),\left(7,6\right),\left(8,4\right),\left(9,5\right). \end{array}$$
The white solid point on the right is the position solution sequence obtained after the replacement operation. At this time, the position solution sequence of the bat is
  (30) $$\begin{array}{c} \left(1,1\right),\left(2,2\right),\left(3,4\right),\left(4,5\right),\left(5,5\right),\left(6,8\right),\left(7,6\right),\left(8,4\right),\left(9,5\right). \end{array}$$
*Step 3*. Delete the repeated position solution of the second component (unique operation). After the remainder operation, the second component of the position solution will have repeated values. At this time, it is time to delete the duplicate position solution.
Using the following formula, the position solution of the deleted second component is repeated, where unique is the deletion function:
  (31) $$\begin{array}{c} x_{i}^{t}=\mathrm{unique}\left(x_{i}^{t}\right). \end{array}$$
The unique operation is shown in Figure 5. The left side is the current position solution sequence:
  (32) $$\begin{array}{c} \left(1,1\right),\left(2,2\right),\left(3,4\right),\left(4,5\right),\left(5,5\right),\left(6,8\right),\left(7,6\right),\left(8,4\right),\left(9,5\right). \end{array}$$
After executing the unique operation, the position solution sequence becomes
  (33) $$\begin{array}{c} \left(1,1\right),\left(2,2\right),\left(3,4\right),\left(4,5\right)\left(6,8\right),\left(7,6\right). \end{array}$$
The deleted location solution is
  (34) $$\begin{array}{c} \left(5,5\right),\left(8,4\right),\left(9,5\right). \end{array}$$
That is, the position solution where the second component is repeated, as shown in Figure 5.
*Step 4*. Fill position solution sequence (fill operation). From the position solution sequence after a unique operation, the algorithm obtains all the first components to form a set FSet. The algorithm obtains all the second components to form the set SSet.

The algorithm obtains a set of random number sequences of the source model face number *m* and finds all the values that do not appear in FS to form the first component set FS_1_. After that, the algorithm obtains a set of random number sequences of the target model face number *n* and finds all the values that do not appear in SS to form the second component set *SS*_1_. From FS_1_ and SS_1_, the algorithm randomly selects a numerical value to form a position solution and adds it to the position solution sequence until FS_1_ and SS_1_ are empty.

The fill operation process is shown in Figure 6, and the left side represents the position solution sequence to be processed:

(35) $$\begin{array}{c} \left(1,1\right),\left(2,2\right),\left(3,4\right),\left(4,5\right),\left(6,8\right),\left(7,6\right). \end{array}$$

The white solid dot on the right represents the new position solution. The transformed position sequence is

(36) $$\begin{array}{c} \left(1,1\right),\left(2,2\right),\left(3,4\right),\left(4,5\right),\left(5,3\right),\left(6,8\right),\left(7,6\right),\left(8,7\right),\left(9,9\right). \end{array}$$

Since the points in the structural similarity matrix between the source model and the target model are all discrete points, when the bat algorithm searches this matrix, the position solution obtained is also discrete. This requires processing these position solutions to reacquire the current optimal position solution sequence. The face matching process based on the bat algorithm is as follows:

*Step 1*. The algorithm calculates the shape similarity and neighborhood structure similarity between the source model surface and the target model surface. Moreover, the algorithm constructs a structural similarity matrix FC between the source model and the target model.
*Step 2*. Initialize the population. The algorithm sets the population size *N*, the number of iterations count, the maximum number of iterations Maxk, the initial loudness *A*_*i*_^0^ of the *i*th bat at the moment *t*=0, the pulse rate *r*_*i*_^0^, and the maximum value *Q*_max_ and minimum value *Q*_min_ of the pulse frequency.
*Step 3*. The algorithm calculates the fitness function value *f*(*i*)(*i*=1,2,…, *n*) of the *i*th bat and obtains the smallest fitness function value *f*_min_ and its corresponding optimal position solution *x*^*∗*^.
*Step 4*. If
  (37) $$\begin{array}{c} \mathrm{count}=\mathrm{Maxk,} \end{array}$$
then the algorithm ends, and the current optimal position solution *x*^*∗*^ is output; otherwise, count++, and the algorithm goes to Step 5.
*Step 5*. The algorithm redefines various values and rounds the speed *v*_*i*_^*t*^ and position *x*_*i*_^*t*^ of the *i*th bat at time *t*.
*Step 6*. The algorithm performs mod processing on *x*_*i*_^*t*^ and judges whether there is a 0 solution in the surface sequence position solution. If there is 0 solution, the algorithm goes to Step 7; otherwise, the algorithm executes Step 8.
*Step 7*. Through the replace operation, the algorithm handles the 0 solution problem in the position solution sequence.
*Step 8*. The algorithm performs unique processing to delete the repeated position solutions in the current surface sequence.
*Step 9*. Through the fill operation, the algorithm handles the empty solution problem in the surface sequence position solution and obtains a new undetermined solution *x*_new_.
*Step 10*. The algorithm generates a random number rand1. If *r* and 1 > *r*_*i*_^0^, the position of the best bat in the current group shifts to the next position, the algorithm goes to Step 6; otherwise, the algorithm goes to Step 11.
*Step 11*. The algorithm generates a random number rand2. If rand2 < *A*_*i*_^0^ and *f*(*x*_new_) < *f*(*i*), then *f*(*i*)=*f*(*x*_new_) and *x*_*i*_^*t*−1^=*x*_new_; otherwise, *f*(*i*) and *x*_*i*_^*t*−1^ do not change.
*Step 12*. If *f*(*x*_*new*_) < *f*_min_, then *x*^*∗*^=*x*_new_; otherwise, *x*^*∗*^ does not make any changes, and the algorithm returns to Step 4.

The bat algorithm is used to search the structural similarity matrix, and the final optimal position solution vector is (*j*(1), *j*(2),…, *j*(*m*)). It can be known that the matching sequence between the source model and the target model is (1, *j*(1)), (2, *j*(2)),…, (*m*, *j*(*m*)).

### 5.4. The Analysis Effect of the Model on Sports Movements

The scientific analysis of sports actions is carried out through the model constructed above, the algorithm in this paper is named HB algorithm, and the algorithm performance of the algorithm proposed in this paper is compared with neural network algorithm (NN) and deep learning algorithm (DL). First, this paper compares the effects of sports action feature recognition and compares 40 sets of actions. The results are shown in Figure 7.

It can be seen from the above chart that the hybrid model constructed in this paper performs well in recognition of sports action features, while the recognition rates of traditional neural network algorithms and deep learning algorithms are low. Next, this paper analyzes the scientific evaluation of the action by the algorithm love, the results are expressed by the scoring method, and the action correction opinions are scored. The results are shown in Figures 8 and 9.

It can be seen from the above figure and table that the algorithm in this paper performs very well in action evaluation and action correction, which is much higher than the traditional algorithm. It can be seen that the algorithm in this paper has a certain effect.

## 6. Conclusion

This paper combines the greedy algorithm and the bat algorithm to construct an intelligent model that can be applied to sports action analysis. Moreover, this paper designs and implements CAD model retrieval methods based on greedy algorithm and bat algorithm. In addition, this paper focuses on the retrieval process based on the greedy algorithm and the bat algorithm and compares and analyzes the advantages and disadvantages of the two algorithms in model retrieval based on experimental data. The results show that the bat algorithm is feasible in model retrieval, and the bat algorithm is better than the greedy algorithm when measuring the subtle differences between CAD models. The pros and cons of the order are used to judge the degree of similarity between the model faces and apply it to the structural similarity matrix between the models. At the same time, this paper establishes the corresponding mathematical model for the shape and structure of the model and constructs the shape similarity matrix, the surface neighborhood structure similarity matrix, and the structure similarity matrix between the source model and the target model. Finally, this paper designs experiments to verify the performance of the model. From the research results, it can be seen that the model constructed in this paper has a certain effect.

## Figures and Tables

**Figure 1:** MapReduce workflow.

**Figure 2:** Flowchart of distributed greedy EM algorithm.

**Figure 3:** Iterative process of distributed greedy EM algorithm.

**Figure 4:** Replace operation.

**Figure 5:** Unique operation.

**Figure 6:** Fill operation.

**Figure 7:** Comparison diagram of the accuracy rate of sports action feature recognition.

**Figure 8:** Comparison diagram of standard evaluation of actions.

**Figure 9:** Comparison diagram of scores of action correction opinions.

## Data Availability

The data used to support the findings of this study are available from the author upon request.
